The article "Study on Risk Factors for Death from Cardiomyopathy and Effectiveness of Health Information Management" was published in 2021. Journal: J Healthc Eng.

# Study on Risk Factors for Death from Cardiomyopathy and Effectiveness of Health Information Management

**DOI:** 10.1155/2021/3922611

**Published:** 2021-12-07

**Authors:** Lei Wang, Shuping Zhang, Yan Wang, Jin Xuan, Yanli Han, Jianlin Ke

**Affiliations:** ^1^Special Inspection Section, The Second Affiliated Hospital of Shandong University of Traditional Chinese Medicine, Jinan, 250001, Shandong Province, China; ^2^Department of Cardiology, The Second Affiliated Hospital of Shandong University of Traditional Chinese Medicine, Jinan, 250001, Shandong Province, China

## Abstract

**Objective:**

To explore risk factors for death from cardiomyopathy and the effectiveness of health information management (HIM).

**Methods:**

A total of 80 patients with cardiomyopathy admitted in ICU of our hospital (January 2016–January 2020) were selected as study subjects, and the clinical data of the patients were retrospectively analyzed. The patients were divided into the survival group (*n* = 72) and the death group (*n* = 14) according to the treatment outcome. Then, according to the management mode, the survival group was further equally divided into the conventional group and the HIM group to investigate the influence of risk factors on prognosis of patients with cardiomyopathy and the effectiveness of HIM.

**Results:**

No significant difference was found in baseline body mass, myocardial enzymes, troponin, infection factors, history of heart disease, and gender between the survival group and the death group (*P* > 0.05). Compared with the survival group, the patients of the death group were older (*P* < 0.05), LVEF of the death group was obviously lower (*P* < 0.05), and the scores of APACHE II and SOFA of the death group were obviously higher (*P* < 0.05). Further logistic regression analysis of the univariate factors influencing the risk of death from cardiomyopathy led to the conclusion that LVEF was an independent risk factor for death in patients with cardiomyopathy. LVEF below 24.69% examined by echocardiography had a high predictive value, with a sensitivity of 98.6% and a specificity of 78.6%. No obvious difference was found in general data between the conventional group and the HIM group (*P* > 0.05). Compared with the conventional group, the disease remission rate, complication rate, awareness rate of health knowledge, ICU length of stay, and scores of self-management efficacy of the HIM group were obviously better (*P* < 0.05). No significant difference was found in 5-year mean survival rate between the conventional group and the HIM group (*P* > 0.05).

**Conclusion:**

Older age, lower LVEF, and higher scores of APACHE II and SOFA are all risk factors for death from cardiomyopathy. Lower LVEF is an independent risk factor, and LVEF below 24.69% is an important indicator of increased risk of death. Moreover, HIM can effectively improve short-term treatment efficacy but has little effect on the long-term survival rate.

## 1. Introduction

Cardiomyopathy is a heterogeneous group of myocardial diseases with the presence of ventricular hypertrophy or dilation, and in severe cases, it can lead to cardiovascular death or progressive heart failure [1–4]. The cause of primary cardiomyopathy is not clear, and that of secondary cardiomyopathy is mostly related to infection, endocrine disease, allergy, and ischemia. Relevant studies have shown that cardiac function can be significantly improved or rehabilitated in some patients within days to weeks, whereas some critically ill patients with severely reduced cardiac function generally die from severe left heart failure or malignant arrhythmias, with left ventricular systolic dysfunction observed by ventriculography [5–8]. At present, cardiomyopathy has been continuously explored in many clinical research studies, but its risk factors for death remain to be further investigated. Therefore, this study will focus on the risk factors for death from cardiomyopathy (such as age, gender, history of heart disease, and relevant clinical indicators). Moreover, most patients with cardiomyopathy gradually return to normal cardiac function after the condition is controlled, so it is vital to ensure their prognostic effect and quality of life. In this way, health information management (HIM) is implemented in our hospital, which has been recognized by many patients. HIM is generated in the context of the new data era, which adapts to the social environment, technological progress, and individualized needs while meeting the medical needs of health management with big data, aiming to improve the level and quality of health management efforts under new circumstances. So this paper aims to further clarify the effectiveness of HIM for patients with cardiomyopathy by carrying out a combined study.

## 2. Materials and Methods

### 2.1. Screening and Grouping of Patients

A total of 80 patients with cardiomyopathy admitted in ICU of our hospital (January 2016–January 2020) were selected as the study subject, and the clinical data of the patients were retrospectively analyzed. The patients were divided into the survival group (*n* = 72) and the death group (*n* = 14) according to the treatment outcome. Then, according to the management mode, the survival group was further equally divided into the conventional group and the HIM group, with 36 cases in each group. The study was approved by the Hospital Ethics Committee.

### 2.2. Inclusion Criteria

The inclusion criteria are as follows: (1) All the patients met the clinical diagnostic criteria of cardiomyopathy in Internal Medicine (7th Edition) [9]. (2) The heart function (New York Heart Association, NYHA) of patients was I–IV. (3) The clinical data of patients were complete. (4) Patients did not have cognitive disorders, communication disorders, and limb activity disorders. (5) Patients did not have history of familial cardiomyopathy. (6) Patients and their families understood the study and signed the consent form.

### 2.3. Exclusion Criteria

The exclusion criteria are as follows: (1) Patients were combined with other organ and tissue lesions or malignant tumors. (2) Patients or their families failed to coordinate with HIM. (3) Patients had poor treatment compliance. (4) The time of follow-up was less than 12 months. (5) Patients had primary cardiomyopathy. (6) Patients were complicated with cardiovascular diseases such as myocardial infarction, heart failure, and valvular heart disease.

### 2.4. Methods

#### 2.4.1. Research Plans of Risk Factors for Death from Cardiomyopathy

The risk factors were analyzed in terms of age, baseline body mass, left ventricular ejection fraction (LVEF), scores of the Acute Physiology and Chronic Health Evaluation (APACHE II) within 24 h of entering the ICU, scores of Sequential Organ Failure Assessment (SOFA), myocardial enzymes, troponin, infection status based on patients' temperature, hemogram, imaging data, bacterial culture, history of heart disease, and gender.

#### 2.4.2. Health Management Intervention

The conventional group was given routine health management. After admission, the doctors and responsible nurses carried out routine health education for the patients and their families and established health management files. The patients were followed up by telephone every week within the first month after discharge (the time was not less than 15 minutes), and then followed up by telephone every month for one year. After one year, the patients were followed up by telephone every 3 months according to their actual situations [10, 11].

The HIM group was given health information management. First, a special group of cardiomyopathy health management composed of doctors and nurses received regular training on health management knowledge about cardiomyopathy medical care. After admission, the patients' condition was comprehensively evaluated, and health management files were established, mainly including general data, disease conditions, contact information, and WeChat number. Secondly, a health management platform was built on WeChat for family members, nursing staff, and medical teams. The platform mainly included medical information, patients' information, and health management. The nursing staff uploaded the health information files of each patient in time, so the platform could prompt the nursing staff to monitor and give intervention to patients timely, which was conducive to the doctors to formulate targeted treatment plans according to the specific conditions of the patients and to supervise the implementation of the plans through the platform [12, 13]. During hospitalization, the patients were diagnosed and treated by medical specialists. After discharge, the nursing staff uploaded all the health education, diagnosis, and treatment information and nursing plans to the information platform, and then the community nursing staff carried out targeted intervention on their health status.

### 2.5. Observation Indexes

According to the study criteria of Maron et al. [14], cardiac function recovery - Grade I indicated disease remission, and the patients' disease remission rate was calculated. The self-made health knowledge questionnaire (referring to the SF-36 scale) was used to evaluate the understanding degree of related diseases, and the awareness rate was calculated (>80% indicated qualified). The range of Cronbach's *α* efficient was 0.63–0.89, and each scale had good discrimination validity, structure validity, and reliability. The self-management efficacy scale [15] was used to evaluate patients' self-management abilities, mainly including daily living and compliance behaviors, with a score of >60 points as qualified. The ICU length of stay and the incidence of complications were also recorded.

### 2.6. Statistical Processing

All statistical data of the study were processed by SPSS22.0 to calculate the difference between groups, and the pictures were graphed by GraphPad Prism 7 (GraphPad Software, San Diego, USA). Including enumeration data and measurement data in the form of [*n* (%)] and ($\bar{x}$ ± *s*), respectively, the study used the *X*^2^ test and *t*-test. The differences were statistically significant at *P* < 0.05.

## 3. Results

### 3.1. Analysis of Risk Factors for Death from Cardiomyopathy

No significant difference was found in baseline body mass, myocardial enzymes, troponin, infection factors, history of heart disease, and gender between the survival group and the death group (*P* > 0.05). Compared with the survival group, the patients of the death group were older (*P* < 0.05), LVEF of the death group was obviously lower (*P* < 0.05), and the scores of APACHE II and SOFA of the death group were obviously higher (*P* < 0.05); see Table 1.

### 3.2. Logistic Analysis of Risk Factors for Death from Cardiomyopathy

Further logistic regression analysis of the univariate factors influencing the risk for death from cardiomyopathy led to the conclusion that LVEF was an independent risk factor for death in patients with cardiomyopathy, as shown in Table 2.

### 3.3. LVEF in Predicting Death for Patients with Cardiomyopathy

LVEF was an independent risk factor for death in patients with cardiomyopathy. LVEF below 24.69% examined by echocardiography had a high predictive value, with a sensitivity of 98.6% and a specificity of 78.6%, as shown in Figure 1 and Table 3.

### 3.4. General Data of the Conventional Group and the HIM Group

The survival group was divided into the conventional group and the HIM group according to management mode. No obvious difference was found between the two groups in general data such as age, BMI, history of heart disease, education degree, and profession (*P* > 0.05), as shown in Table 4.

### 3.5. Short-Term Efficacy of HIM

Compared with the conventional group, the disease remission rate, complication rate, awareness rate of health knowledge, ICU length of stay, and scores of self-management efficacy of the HIM group were obviously better (*P* < 0.05) (Table 5).

### 3.6. Long-Term Efficacy of HIM

The mean follow-up time of the conventional group was (61.55 ± 3.26) months and that of the HIM group was (61.83 ± 3.31) months, without any obvious difference between both groups (*t* = 0.362, *P* = 0.719). In addition, no significant difference was found in the 5-year mean survival rate between the conventional group and the HIM group (*P* > 0.05)(Figure 2).

## 4. Discussion

Cardiomyopathy is an organic disease with the presence of abnormal mechanical activity of the heart or electrocardiogram dysfunction, which can affect the systolic and diastolic functions of the heart and even lead to severe heart failure, atrial or ventricular arrhythmia, and embolism in severe cases. At present, the pathogenesis of most cardiomyopathies remains unclear. Besides genetic factors, inflammation, infection, immune dysfunction, endocrine, and metabolic abnormalities are also common pathogenic factors. In addition, cardiomyopathy in some patients is associated with tachycardia, abnormal protein deposition of myocardial interstitium, and left ventricular myocardial densification [16, 17]. Cardiomyopathy has high mortality rates, but there are few reports on the analysis of risk factors for death in China. Moreover, a large number of clinical reports have shown that most patients with cardiomyopathy have a poor prognosis, which is mainly determined by the patients' left ventricular function and hemodynamics, with a 5-year survival rate of only 50% and a 10-year survival rate of about 25%, according to authority data. However, with the development of diagnosis and treatment, the 5-year survival rate of patients has been up to 65.5–75% [18–20]. Therefore, with the help of advanced health management concepts, the health industry in China will embrace more rapid development. However, at present, China's health management is still in the primary stage, and there are many problems to be solved. Therefore, an innovative service system and operation mode of health management with Chinese characteristics need to be established. Moreover, most patients with cardiomyopathy have a poor prognosis, and according to authority data, their 5-year survival rate is only 50%, and such patients usually require close observation of left ventricular function and hemodynamics. Hence, it is necessary to introduce HIM to them. Based on the above, this paper explored risk factors for death from cardiomyopathy and the effectiveness of HIM, and by combining with patients' clinical manifestations and relevant study results, included factors such as patients' baseline body weight, myocardial enzyme, troponin, infection factors, history of heart disease, gender, age, and APACHE II scores and SOFA scores into the analysis on risk factors for cardiomyopathy.

The study showed that no significant difference was found in baseline body mass, myocardial enzymes, troponin, infection factors, history of heart disease, and gender between the survival group and the death group (*P* > 0.05). Compared with the survival group, the patients of the death group were older (*P* < 0.05), LVEF of the death group was obviously lower (*P* < 0.05), and the scores of APACHE II and SOFA of the death group were obviously higher (*P* < 0.05). Norrishgabrielle et al. [6] reported that over 75 years old was an independent risk factor of death from cardiomyopathy. In this study, the mean age of the death group was 71.15, while that of the survival group was 62.41, which may be attributed to that an older age was inclined to reduced cardiac function, so poor compensatory capacity was one of the important reasons for increased mortality risk. As reported in BAZOUKIS [21], a significant decrease in LVEF at onset is also an independent risk factor for death from cardiomyopathy, which is consistent with this study. The scores of APACHE II and SOFA can reflect the comprehensive symptoms of severe patients, which has a positive effect on the prognosis of patients. Meanwhile, the scores of APACHE II and SOFA of the death group were significantly higher, indicating that the death group had a severer disease. Further logistic regression analysis of the univariate factors influencing the risk of death from cardiomyopathy led to the conclusion that LVEF was an independent risk factor for death in patients with cardiomyopathy. LVEF below 24.69% examined by echocardiography had a high predictive value, with a sensitivity of 98.6% and a specificity of 78.6%. After further analysis, the causes of death may be depressed cardiac systolic function and cardiogenic shock, which is followed by cardiac ischemia and even a higher risk of coronary thrombosis. With deep sedation and muscle relaxants, the patients' oxygen consumption was markedly reduced. Meanwhile, patients' intake and output were closely monitored and were maintained at a comparatively low volume load. In this way, with LVEF below 30%, the cardiac systolic function can be recovered within one week for many patients, and when it drops to less than 24.69%, the cardiac compensatory capacity is severely reduced. Therefore, the above measures fail to work on acute left heart failure, which eventually results in a higher risk of death for patients.

Compared with the conventional group, the disease remission rate, complication rate, awareness rate of health knowledge, ICU length of stay, and scores of self-management efficacy of the HIM group were obviously better (*P* < 0.05). No significant difference was found in the 5-year mean survival rate between the conventional group and the HIM group (*P* > 0.05). Health management Informatics is an inevitable choice for improving the efficiency and quality of health management services, with the purpose of reducing costs and optimizing services. It is a new opportunity brought by the Internet's development, which not only enriches the communication method but also greatly improves the management efficiency with the support of big data [22–24]. With more comprehensive content and more coordinated business, this mode enables convenient online health management through more precise monitoring of long-term dynamic information and emphasizes patients' self-management. The results of this study suggest that HIM can effectively improve the incidence of complications in patients with cardiomyopathy, help to control the disease, and enhance the self-management efficacy and their quality of life, but HIM has little impact on the long-term survival rate according to statistical data, which may be due to the small sample size in this study, so it is still necessary to confirm that by expanding the sample size and carrying out multicenter research. In addition, the study was a retrospective analysis study with some limitations. For example, analysis of single factors affecting cardiomyopathy could only be conducted according to the existing situation, and other risk factors could not be preset. Therefore, subsequent related research should comprehensively analyze the risk factors affecting cardiomyopathy via prospective studies and preset the study process by combining with the existing research results.

To sum up, older age, lower LVEF, and higher scores of APACHE II and SOFA are all risk factors for death from cardiomyopathy. Lower LVEF is an independent risk factor, and LVEF below 24.69% is an important indicator of increased risk of death. Moreover, HIM can effectively improve short-term treatment efficacy but has little effect on the long-term survival rate.

## Figures and Tables

**Figure 1:** ROC curve.

**Figure 2:** 5-year survival rate (%).

**Table 1:** Analysis of risk factors for death from cardiomyopathy.

Indexes	Survival group	Death group	*X* ^2^/*t*	*P*
Age (years)	62.41 ± 11.26	71.15 ± 15.82	4.174	<0.001
Baseline body mass (kg)	61.94 ± 10.05	62.11 ± 10.08	0.111	0.912
LVEF (%)	32.01 ± 3.61	23.17 ± 2.04	8.863	<0.001
APACHEII	15.14 ± 2.32	19.05 ± 3.31	5.357	<0.001
SOFA score	7.38 ± 2.14	10.01 ± 3.19	3.858	0.002
Myocardial enzymes (*μ*/l)	31.74 ± 4.60	32.05 ± 4.55	0.444	0.657
Troponin (ng/ml)	0.12 ± 0.05	0.13 ± 0.04	1.448	0.149
Infectious factors			2.573	0.109
Infected	40 (55.56)	11 (78.57)		
Uninfected	32 (44.44)	3 (21.43)		
History of heart disease			2.273	0.132
Y	25 (34.72)	2 (14.29)		
N	47 (65.28)	12 (85.71)		
Gender			0.293	0.588
Male	26 (36.11)	4 (28.57)		
Female	46 (63.89)	10 (71.42)		

**Table 2:** Logistic analysis of risk factors for death from cardiomyopathy.

Variable	*B*	S.E.	Wals	*df*	Sig.	Exp (*B*)
Age	−0.066	0.038	3.421	1	0.064	0.936
LVEF	−0.704	0.210	11.204	1	0.001	0.495
APACHEII	0.048	0.122	0.157	1	0.692	1.050
SOFA score	−0.050	0.046	3.214	1	0.071	0.951

**Table 3:** Area under the curve.

Area	Standard error^a^	Asymptotic sig.^b^	Asymptotic 95% confidence interval	
			Lower limit	Upper limit
0.985	0.012	0.000	0.000	1.000

“a” indicated under nonparametric assumptions; “b” indicated zero hypothesis; real area = 0.5.

**Table 4:** Comparison of general data between the two groups (*n* = 36).

Observation indexes	Conventional group	HIM group	*X* ^2^/*t*	*P*
Age (years)	58.94 ± 6.28	59.16 ± 6.41	0.147	0.884
BMI (kg/m^2^)	23.11 ± 3.25	23.27 ± 3.31	0.207	0.837
Gender			0.056	0.813
Male	16 (44.44)	17 (47.22)		
Female	20 (55.56)	19 (52.78)		
History of heart disease			0.348	0.555
Y	2 (5.56)	1 (2.78)		
N	34 (94.44)	35 (97.22)		
Education degree			0.225	0.635
Middle school degree and below	21 (58.33)	19 (52.78)		
Junior high school degree and above	15 (41.67)	17 (47.22)		
Occupation				
Civil servant	6 (16.67)	8 (22.22)	0.355	0.551
Teacher	4 (11.11)	5 (13.89)	0.127	0.722
Farmer	13 (36.11)	15 (41.67)	0.234	0.629
Retiree	7 (19.44)	4 (11.11)	0.966	0.326
Others	6 (16.67)	4 (11.11)	0.466	0.496

**Table 5:** Comparison of short-term efficacy.

Evaluation indexes	Conventional group (*n* = 36)	HIM group (*n* = 36)	*X* ^2^/*t*	*P*
Disease remission rate	13 (36.11)	26 (72.22)	9.455	0.002
Incidence of complications	14 (38.88)	3 (8.33)	9.318	0.002
Awareness rate of health knowledge	21 (58.33)	32 (88.89)	8.651	0.003
ICU length of stay (d)	8.85 ± 2.17	6.90 ± 1.52	4.416	<0.001
Self-management efficacy	77.12 ± 13.54	62.78 ± 12.05	4.747	<0.001

## Data Availability

Data used to support the findings of this study are available on reasonable request from the corresponding author.
